RETRACTED

# Improved Giza pyramids construction algorithm for Modify the deep neural network-based method for energy demand forecasting

**DOI:** 10.1016/j.heliyon.2023.e20527

**Published:** 2023-09-29

**Authors:** Xue Wang, Saeid Razmjooy

**Affiliations:** a Admissions and Employment Guidance Center, Xi'an Peihua University, Xi'an 710125, Shaanxi, China; b Department of Engineering, University of Mohaghegh Ardabili, Ardabil, Iran; c College of Technical Engineering, The Islamic University, Najaf, Iraq

**Keywords:** Energy demand, Forecasting, Deep neural networks, Efficiency, Improved giza pyramids construction algorithm

## Abstract

Accurate prediction of energy demand is crucial for improving services, reducing costs, and optimizing operations in energy systems. Deep neural networks (DNNs) have emerged as a popular method for energy demand forecasting. However, the performance of DNNs can be affected by data quality and hyperparameter selection. To address these concerns, this study proposes a novel energy demand forecasting technique that combines DNNs with an enhanced Giza pyramid construction methodology. The aim of this study is to provide a more reliable and effective approach for forecasting energy demand. The DNNs are employed to capture the complex relationships between input and output variables, while the Giza pyramids algorithm is utilized to optimal selection of hyperparameters of the network. Real-world energy demand data is used to evaluate the proposed approach, comparing it with state-of-the-art baseline models. The research methodology involves assessing the suggested approach using real-world energy demand information and conducting a comparative analysis with cutting-edge baseline models, including modified BP neural network (MBPNN), Neural Network based Genetic Algorithm (NNGA), and reinforcement learning and deep neural network (RLDNN). The IGPCA/CNN method outperforms other methods in energy prediction accuracy across short-term, medium-term, and long-term time scales. It achieves an MSE score of 0.564, lower than MBPNN, NNGA, and RLDNN. In medium-term prediction, it achieves an MSE score of 0.587, better than MBPNN, NNGA, and RLDNN. In long-term prediction, it achieves an MSE score of 0.629, lower than MBPNN and RLDNN. Further analysis and validation experiments are needed to ensure robustness and generalizability. Comparing the method with other state-of-the-art approaches can provide a comprehensive understanding of its superiority. The performance of the models is evaluated based on reliability and effectiveness in energy demand forecasting. The major conclusion of this study is that the proposed approach outperforms the initial models in accurately forecasting energy demand. The combination of DNNs and the improved Giza pyramid construction methodology results in enhanced performance, demonstrating superior reliability and effectiveness compared to other models. The study highlights the significance of accurate energy demand prediction for optimizing energy systems and reducing costs.

RETRACTED

## 1 Introduction

The term 'energy demand' refers to the quantity of energy required to fulfill consumer, residential, commercial, and industrial needs [3]. Determining the energy value that must be generated, transferred, and distributed is crucial for the design and operation of energy systems [27]. Accurate energy demand prediction is essential for efficient and reliable operation in energy systems [5]. It enables energy businesses to optimize their operations, reduce costs, and provide higher-quality services [36]. Energy consumption is influenced by various factors such as population growth, economic expansion, energy prices, weather conditions, and technological advancements [6]. To meet the increasing demand while ensuring environmental sustainability and energy security, the energy sector needs to utilize diverse energy sources and technologies, including sustainable energy sources and energy storage systems [13]. Energy businesses also need to invest in advanced forecasting methodologies for energy consumption to streamline their processes and reduce costs [28].

The accurate and energy systems operation depends on the ability to predict energy demand. Energy companies may optimize production, transmission, and distribution operations, lower costs, and boost service quality with the aid of accurate forecasts [32]. Traditional approaches for energy consumption prediction rely on statistical models, which have limitations in identifying complex patterns in data and require extensive feature engineering [21].

In recent years, neural networks (NNs) have demonstrated high potential for energy consumption prediction by automatically extracting features from raw data and capturing intricate relationships between input and output variables. However, achieving optimal performance with NNs depends on balancing input data, adjusting hyperparameters, and optimizing the training process [15]. Training NNs can be computationally expensive, especially when dealing with large datasets [37]. Several methods, such as preprocessing techniques, network structure design, optimization algorithms, and ensemble strategies, have been proposed to address these challenges and improve the accuracy and effectiveness of NNs for electricity demand forecasting [35].

The design of the network architecture is another critical factor affecting the effectiveness of NNs for energy demand forecasting [20]. The choice of network architecture depends on the forecasting objective and the characteristics of the input data [34]. During the training process, optimization algorithms are used to determine the optimal weights and biases for the network variables [11]. Gradient descent techniques, such as stochastic gradient descent, utilize the gradient of the loss function to update the network's variables [14]. Adaptive learning rate approaches like the Adam optimizer can enhance the convergence rate and stability of the training process by dynamically adjusting the learning rate based on the loss function gradient [2].

RETRACTED

The utilization of NNs for energy demand forecasting has shown promising results in enhancing the effectiveness and reliability of energy systems [1]. However, the performance of NNs is influenced by various factors, including data preprocessing, network architecture selection, and training procedures [16]. Energy businesses need to leverage cutting-edge techniques such as data preprocessing, network architecture design, optimization algorithms, and ensemble methods to maximize the benefits of NNs in energy demand forecasting [12]. Recent studies have demonstrated that NNs outperform traditional statistical models in energy consumption forecasting due to their ability to automatically extract features from raw data and capture complex correlations between input and output variables [29]. For example, Long Short-Term Memory (LSTM) neural network proposed by Cheng et al. [7]. They introduced a reduction in predicting error of 21.80% and 28.57%, respectively. Additionally, they demonstrated that metering/forecasting granularity performed once every 30 min can produce greater accuracy compared to other feasible granularity options. The research does not specifically address the potential constraints or drawbacks of the suggested approach. Nevertheless, there exist several possible constraints associated with the utilization of LSTM neural networks for power demand forecasting. These limits include the need of a substantial volume of data to adequately train the model, the potential risk of overfitting, and the computational intricacy inherent in the model. Furthermore, it is important to note that the research only relies on a publicly available dataset, which raises concerns about the generalizability of the findings to other datasets or real-life situations.

Bunnoon et al. [4] conducted a study on mid-term load prediction using the statistical approaches of multiple linear regression (MLR) and autoregressive integrated moving average (ARIMA) methods. The results obtained from their research indicated that the neural network methods outperformed the MLR approach in terms of accuracy. It was found that the performance of neural networks is influenced by the quality of the input data and the selection of hyperparameters, which can have varying effects on the overall performance. However, there are some limitations to this work. Firstly, the study only focused on mid-term load forecasting for Thailand, and the results may not be generalizable to other countries. Secondly, the accuracy of the forecasting models may be affected by unforeseen events such as natural disasters or economic crises. Finally, the study did not consider the impact of renewable energy sources on load forecasting, which could be an important factor in future research.

RETRACTED

To enhance the network architecture in this context, various optimization strategies have been proposed. The utilization of these methodologies for electricity demand prediction can lead to more satisfactory results and improved performance. For example, Liu et al. [22] suggested utilizing a multi-layer perceptron neural network to estimate electrical consumption and freshwater generation in a solar-assisted seawater greenhouse system. According to the findings, the BBO and the GA approaches reduced testing error. Water usage evaluation shows that the ACO technique had the lowest error rate. It was discovered that by changing the width and transparency, increased water production was associated with the ES and GA approaches, with around 120 m3/day and 105 m3/day, respectively. Furthermore, ES, ACO, and GA consume less power. Finally, it was discovered that when the transparency was 0.4, the water production value could be 115 m3/day, whereas when the transparency was 0.6, the value was 95. The experimental results showed that the optimal methods achieved better performance than the traditional LSTM model and neural networks model. However, the optimization methods had weakness such as Getting stuck in local optimization that can reduce the accuracy of optimization methods.

A Deep Neural Network was suggested by Wen et al. [33] to predict electricity demand in the energy industry at the level of individual buildings for a sustainable economy and to minimize pollution in the atmosphere. The results of the study demonstrated that it is possible to forecast 98.1%, increase at 96.8%, satisfy 98.5% of the demand for electricity, consume 97.6% of the available electricity, and have a 96.2% renewable energy ratio which reached superior. The paper does not explicitly mention the limitations of this work. However, some potential limitations could include the need for a large amount of data to train the DNN, the possibility of errors in the data used for training, and the difficulty of accounting for all relevant factors that may impact energy demand. Additionally, the paper focuses on energy demand forecasting at the individual building level, and it may not be directly applicable to larger-scale energy planning and policy-making.

RETRACTED

Dieudonné et al. [10] proposed a hybrid model of artificial intelligence and statistical methods for hourly forecasts of electricity demand over a period of one week in the city of Yaoundé, Cameroon. The model was designed from an optimization algorithm and combined the best parameters of artificial neural networks, multiple linear regression, and Holt exponential smoothing models. The results showed that the proposed hybrid model outperformed most similar models in the literature on the subject, obtaining statistically significant precision values. However, the limitations of this work included the fact that the study was limited to the city of Yaoundé and may not be generalizable to other regions or countries. Additionally, the study only considered short-term forecasting and did not address long-term forecasting.

This research work presents a strong contribution in the field of energy demand forecasting by introducing an improved approach that incorporates a hybrid architecture of Deep Neural Networks (DNNs). The novelty of this study lies in its utilization of the latest advancements in optimization techniques for deep learning, specifically the application of the Improved Giza Pyramids Construction Algorithm (IGPCA).

One key aspect of novelty in this research is the use of DNNs, which are known for their ability to capture complex patterns and relationships in large datasets. By implementing a hybrid architecture of DNNs, the proposed approach harnesses the power of deep learning to provide more efficient and accurate energy demand forecasts. This is crucial in meeting the increasing challenges of energy demand management and load forecasting in today's dynamic energy landscape.

The introduction of the IGPCA further enhances the optimization process in the DNNs used for energy demand forecasting. The IGPCA algorithm improves stability and convergence speed, addressing common issues encountered in training deep neural networks. This novel utilization of the IGPCA algorithm contributes to the overall effectiveness of the proposed approach, providing more robust and reliable energy demand forecasts.

Another significant contribution of this research lies in the focus on handling complex patterns in energy demand data. As consumer behaviors and external factors influence energy consumption, accurately capturing these intricate patterns becomes increasingly important. By incorporating advanced optimization techniques and deep learning methodologies, this study tackles the challenge of understanding and forecasting complex energy demand patterns in a more efficient manner.

RETRACTED

Additionally, the emphasis placed on utilizing up-to-date and high-resolution data further enhances the novelty and relevance of this research. By collecting input and goal data every 20 min from the client end, the proposed approach capitalizes on the timeliness and richness of the dataset used for training the neural network. This approach not only improves the precision of energy usage estimates but also ensures that the forecasted results align closely with real-time consumption patterns.

In summary, this research work offers a valuable and novel contribution to the field of energy demand forecasting. The hybrid architecture of DNNs, coupled with the integration of the IGPCA algorithm, provides an improved approach that addresses the challenges of accurate and efficient energy demand forecasting. By focusing on complex patterns in energy consumption behavior and utilizing up-to-date, high-resolution data, this study enhances our understanding of energy dynamics and supports effective energy management and planning decisions.

## 2 Convolutional neural networks

The present study uses an optimized version of a Convolutional neural network (CNN) to provide an accurate Energy Demand Forecasting. Convolutional neural networks are a form of neural networks that has proven very effective in handling data mining and computer vision challenges. The name “convolutional” is derived from the mathematical action of convolution, which serves as the foundation of these networks. A CNN's architecture is made up of numerous layers, each of which plays a distinct role. The first layer is often a convolutional layer that extracts features from the input picture using filters.

This layer produces a series of feature maps, each of which reflects the reaction of a specific filter to the incoming data. The following layers can be convolutional, pooling, or fully connected, and perform various actions on the input data. The last layer is generally a completely linked layer that generates the network's ultimate output.

A CNN's architecture is made up of numerous layers, each of which plays a distinct role. The first layer is often a convolutional layer that extracts feature from the input data using filters. This layer produces a series of feature maps, each of which reflects the reaction of a specific filter to the incoming data. The following layers can be convolutional, pooling, or fully connected, and perform various actions on the input data. The last layer is generally a completely linked layer that generates the network's ultimate output.

RETRACTED

Convolution layer is the top layer. Data processing frequently employ the linear convolution layer procedure. Convolution is used in CNNs to take features out of an input data. A tiny window, referred to as a kernel or filter, is dragged across the input picture during the convolution procedure, and the dot product between the kernel and the corresponding pixel values in the image is computed. The outcome of this operation is a single value that denotes the filter's activation at that specific point in the data. The convolutional layer may extract distinct characteristics from the input data by using a variety of filters.

Pooling is a down sampling procedure that lowers the feature maps' spatial resolution [26]. Max pooling, which chooses the highest value inside a window and discards the remainder, is the most used pooling procedure. Max pooling is used to provide the network some translational invariance, which allows it to identify the same pattern even if it appears in a different part of the data.

To provide nonlinearity to the network, which is necessary for simulating intricate interactions between the input and output variables, activation functions are utilized. Rectified Linear Unit (ReLU), the most popular activation function in CNNs, converts all negative values to zero while maintaining positive values [30]. Because ReLU is computationally effective and does not have the issue with vanishing gradients, it is preferred over other activation functions like sigmoid and hyperbolic tangent. This unit can be mathematically defined as follows (equations [[1], [2], [3], [4], [5], [6], [7], [8], [9], [10], [11], [12], [13], [14], [15], [16], [17], [18], [19], [20], [21], [22]]) [19]:

(1) f(x)=max(x,0)

When establishing the convolution to add up the dot product and the weights, sliding window is used as a vector and max pooling is used to reduce the output scale. The following layer of the sliding grid in this case has the greatest value. Forward propagation and backpropagation are the two key processes in the CNN training process. The input data is supplied into the network during the forward propagation stage, and the output is generated by spreading the activations through the layers. The gradients of the error with respect to the network parameters are determined using the chain rule in the backpropagation stage. The gradient descent method is used for minimization in this study's backpropagation-based minimizing technique. This may be expressed numerically as follows:

(2) $$L=\sum_{j=1}^{N}\sum_{i=1}^{M}-D_{j}^{\left(i\right)}\;\log\;Y_{j}^{\left(i\right)}$$

where, $D_{j}=\left(0,...,0,\underset{k}{\underbrace{1,\ldots ,1}},0,...,0\right)$ specifies to a vector with suitable output and $Z_{j}$ indicates the $m^{th}$ class of the “Softmax function” which can be defined as follows:

(3) $$Y_{j}^{\left(i\right)}=\frac{e^{f_{j}}}{\sum_{i=1}^{M}e^{f_{i}}}$$

where, M determines the samples number.

RETRACTED

Afterward, by reducing the weight penalty with a coefficient ζ and improving the fitness function,

(4) $$L=\sum_{j=1}^{N}\sum_{i=1}^{M}-D_{j}^{\left(i\right)}\;\log\;Y_{j}^{\left(i\right)}+\frac{\zeta }{2}\sum_{K}\sum_{L}W_{k,l}^{2}$$

where, $W_{k}$, K, and L describe the connection weight, the layer *l* connection quantity and total number, respectively.

By considering the above assumptions, the network error can be achieved as follows:

(5) $$E=\frac{1}{N}\sum_{i=1}^{N}\sum_{j=1}^{k}{\left(D_{ji}-O_{ji}\right)}^{2}$$

where, k, N, $D_{ji}$, and $O_{ji}$ describes the output layers quantity, the training samples, the CNN output, and the correct output, respectively.

The network parameters are then updated using the gradients and an optimization technique like classic optimization algorithms (Adam and stochastic gradient descent (SGD)) or metaheuristics. Metaheuristics do not need explicit knowledge of the issue or gradient information, in contrast to traditional optimization techniques. Instead, they use heuristics to look for answers. Utilizing metaheuristics has the benefit of avoiding local optima, which can be a problem with more conventional optimization techniques like gradient descent.

This is due to the fact that metaheuristics frequently look at a wider search area and can uncover a wider range of solutions. The capacity of metaheuristics to handle complicated and non-linear objective functions, which is typical in CNN training, is another benefit of its use. This is due to the fact that metaheuristics are adaptable and may be used to solve many problems. In contrast to more traditional optimization techniques like Adam or SGD, metaheuristics can be computationally costly and may demand more time and resources. Furthermore, the parameters chosen and the issue being solved may have an impact on how well a metaheuristic performs.

A newly updated metaheuristic algorithm is proposed to give an effective prediction, which may minimize the error between the actual output and the estimated output by varying the internal weights. Overfitting, which happens when the network performs well on the training data but badly on the test data, will be avoided by this regularization. During training, Dropout randomly removes part of the neurons, forcing the network to pick up more reliable characteristics. Weight decay increases the loss function's penalty term, encouraging the network to learn smaller weights and lowering the model's complexity.

RETRACTED

The improved Giza pyramids construction algorithm is used in this work to achieve this. The primary contribution is the application of the improved Giza pyramids construction algorithm to choose the most appropriate number of hyper-parameters for CNN's energy demand forecasting. The lower range and higher range are set to 2 and equal to the size of the sliding window, respectively, to prevent system errors. The minimum amount is chosen since it is the minimum size that is permitted for maximum pooling. Additionally, the amount of the sliding window that needs to be less than the data input is regarded as the problem's inequality constraint. Here, the convolutional neural network's weights, biases, and other parameters are defined as follows:

(6) $$W=\left[w_{1},w_{2},...,w_{p}\right]$$

(7) $$A=\left[a_{1},a_{2},...,a_{A}\right]$$

(8) $$w_{n}=\left[w_{1n},w_{2n},...,w_{\mathrm{Ln}}\right]$$

(9) $$\begin{array}{c} b_{n}=]b_{1n},b_{2n},...,b_{\mathrm{Ln}}]\\ l=1,2,...,L\\ n=1,2,...,N \end{array}$$

where, L, N, l, n, and $w_{in}$ represent, in turn, the total layers' number, the total candidate number, the layer index, the model population number, and the weight number at layer i.

In the following, a comprehensive explanation of the improved Giza pyramids construction algorithm has been described.

## 3 Improved giza pyramids construction algorithm (IGPCA)

### 3.1 Giza pyramids construction optimizer (GPCO)

The Giza Pyramids (Giza Necropo-lis) is a location with 3 enormous pyramids that were constructed when the 4th dynasty in Egypt governed. Based on the information of archaeology, the erection method of these 3 pyramids is different on the grounds that they have been erected during time. The workers' management was considered the most overarching issue in the erection process of pyramids. The optimized pyramids' erection has been important because of hardware amenities’ shortage, limited and short time of erection, and the considerable quantity of utilized blocks of stone. The method of erection, the motivation, and the offered optimizer have been explained in the following.

### 3.2 The erection method

There is the vast array of theories about the erection methods of pyramids. Most archeologists are of the opinion that the pyramids’ stones were gained from mines, transported to the site and finally placed with ramps for mounting the huge stones to the higher places. The Greeks opined that slaves worked hard and they were abused in the erection of pyramids; new excavations, however, clarify that the builder of such constructions were workers with high skills and they all lived in the adjacent villages. The required human sources for erection of the pyramids were between 14000 and 40000 who worked on the range of [10–20 years] for the erection without facilities and tools.

RETRACTED

Beside the construction difficulties, such buildings process needed a progressive tactic for erection management, and issues like workers’ housing, food, salary, and time scheduling. The logistical needs and complication of this project have been extraordinary in retrospect.

### 3.3 The motivation

The workers of the pyramids were considered a combination of slaves and skillful persons who were led by an expert. This proficient manager is named Pharaoh's distinct agent who supervised the process of stone carrying by different workers. The workers should report the tasks implementation to Pharaoh's distinct agent who has the finest rank in group. Every worker owns a specific position (rank) at the site which can be promoted in a way that whenever a worker performs well, he is ranked as a sublime. Accordingly, a competition exists amid workers for getting this rank. What is more, workers might need some rest because of their energy loss over the stones' carrying. Thus, the tired workers is going to be replaced with a new and energetic ones. It shows that if any improvement no longer exists in the human sources, they must be replaced because they could be effective in another place. It implies that there is also another confliction among workers rather than gaining sublime rank; this competition motivates each worker to become experienced and expertise.

Throughout the process of pyramid erection, miners scatter the stone blocks which are to the site by workers. The collecting and carrying of the stone blocks are implemented on regular basis. Although ramps were utilized in the erection of the pyramids, the blocks must be carried to its installation situation. This distance (among stone blocks and its installation state) is determined via the workers’ capability. Workers will carry more and more stones to the installation location if they have enough amount of power that makes the stones far closer to the pyramid erection site. It is of primary importance to note that the motion of stone blocks has been influenced by the primary speed, force of friction, and the gradient of ramp.

### 3.4 The offered optimizer

We assume that there are the stone blocks around the erection site of pyramid, and these stones have to be pushed by the workers to the site. For each stone block, we have its 1st situation and objective function value. As ramps have been utilized for moving the stones to the site, the motion of blocks have been effected by the ramp's friction impact and slope. What is more, the workers frequently move for finding the finest place to control the block. Due to the fact that every worker has different features, there is the probability of substituting workers to strike a balance among the workers' power. Thus, some workers' will be replaced with other ones. Such a replacement leads to an alteration in the power balance and the stone block moving. Some principles exist for the offered optimizer which are described as below.

1. A ramp which is straight-on has been utilized in the pyramid erection.
2. Just one ramp is considered to be utilized.
3. In the algorithm, if the ramp angle with horizontal axis is considered ∅, in the offered optimizer ∅<15° and it can vary. (Based on archaeologists opinion, 8°<∅<12°).
4. As the blocks are really pushed by the workers, solutions have been gained from the block and worker situation resultant.
5. Friction is no longer assumed for workers, but it impacts the stone block displacement.
6. Some workers might be replaced and located in a new situation over the process of erection.

RETRACTED

Some equations are required for an item (stone block) motion on the ramp. As the item makes movement along the ramp, we change the coordinate axis in a way that the x-axis direction and the acceleration direction become the same. Subsequently, the applied force to the block is no longer vertically and horizontally, and the mass force (mg) is located on the axis. Based on the principle of optimizer, every block has been pushed upward on the ramp with the speed of $v_{0}$. Hence, the block does stop after navigating the d space on ramp. 3 forces have been applied to the block, mgsin∅, mgcos∅ , and $f_{k}$ which is the force of kinetic friction. Whenever the block is settled at the displacement threshold, $f_{k}$ could be gained as below based on the formula of max force of static friction:

(10) $$f_{k}=\mu_{k}mgcos\emptyset$$

Here $\mu_{k}$ signifies the coefficient of kinetic friction, m and g illustrate the block mass and the earth gravity (g=9.8), and ∅ is the angle of ramp with the horizontal axis. On the basis of the 2nd low of Newton we have the below formulation on the x-axis:

(11) $$-mgsin\emptyset -f_{k}=ma$$

In the above formula the block acceleration has been shown by a which direction on the ramp is upward and it can be gained by the below formula:

(12) $$a=-g\left(\sin\emptyset +\mu_{k}\;\cos\emptyset \right)$$

There is a need for a motion formula which is no longer depended on the when the acceleration is constant. Such a formula for calculating the block motion could be gained based on the below formula:

(13) $$d=\frac{v_{0}^{2}}{2g\left(\sin\emptyset +\mu_{k}\;\cos\emptyset \right)}$$

Here the displacement value is demonstrated by d. ∅ and $v_{0}$ demonstrate the ramp angle with horizon and the stone initial speed. It is important to note that $v_{0}$ is computed via a random number which is distributed uniformly in every epoch. According to this explanations, the block does start its moving with the velocity of $v_{0}$ providing that a worker does apply power to a block. Based on physics, the block stops moving after a chunk of time because of the friction force. For that reason, another force is applied on the block by the worker which causes the block to start its movement with $v_{0}$. As mentioned, $v_{0}$ has been assumed a random amount over every epoch on the grounds that the applied power for moving the block does vary regarding the consumed power by the worker. Therefore, $v_{0}$ is a random amount between zero and one that can be formulated based as below:

(14) $$v_{0}=\begin{array}{cc} random\left(0,1\right) & 0<random\left(0,1\right)<1 \end{array}$$

What is more, $\mu_{k}$ can be determined using a random amount that is distributed uniformly on the grounds that the surface of ramp is not completely. The reason for the randomness of the amount of friction is that the ramp surface is not completely scrubbed and the friction might reduce or increase because of the potential roughness on the ramp. Therefore, $\mu_{k}$ could be calculated as below:

(15) $$\mu_{k}=\begin{array}{cc} random\left(\mu_{k,l},\mu_{k,h}\right) & \mu_{k,l}<\mu_{k}<\mu_{k,h} \end{array}$$

Here $\mu_{k,l}$ and $\mu_{k,h}$ are the lowest and the highest value of friction coefficient have been predetermined in the offered algorithm, then, in every epoch, a random amount among them is considered. Regarding the main idea of the optimizer, the workers who push the blocks regularly shake or make a movement for controlling the block well. Such shocks provide non-repetitive movements performance of workers for pushing the block well.

RETRACTED

For obtaining the updated situation of the worker, we can utilize the formula which is previously used for calculating d. This formula is employed with little alteration for determining the worker renewed location. When it comes to the worker the friction is no longer assumed. Hence, the renewed location for a worker who pushes the block can be gained using the below formula:

(16) $$y=\frac{v_{0}^{2}}{2gsin\emptyset }$$

y signifies the movement value of the worker regarding its previous location. The worker keeps moving in an upward direction with the block and in the same time does apply power to block. The worker makes tiny movements during pushing the block because he sets his goal on controlling the block well. Due to the fact that there is an initial speed for the workers, the friction force is no longer assumed for him. Such a consideration is one principle of the optimizer that is mentioned earlier. Having determined the alterations in the block and worker movement using the above formulas, a new location could be gained which is assumed a new result for the optimizing problem. For obtaining the new result we have:

(17) $$\vec{l}={\vec{(l}}_{i}+d)\times y{\vec{\sigma }}_{i}$$

Here, d, y, and ${\vec{l}}_{i}$ determine the values of block displacement, worker movement, and the existing location of the block, respectively. ${\vec{\sigma }}_{i}$ signifies a random vector regarding the Lévy distribution. Accordingly, the new location has been attained via adding the earlier location to the block displacement, multiplied by the worker displacement value. Having multiplied this factor, we can determine the worker situation around the block for the forthcoming epoch. Throughout the pyramids’ erection, the worker sometimes becomes tired and lose his ability/power and he is going to be replaced by the other worker. Such a replacement is for power balancing. Having done it, each worker is employed for pushing the appropriate block based on his capability. Thus, a worker with low effectiveness in his vacation might perform far better in another vacation. This process is executed in the optimizer with the probability of 50% (by default). Accordingly, a chance of being replaced for one worker is fifty percent over every epoch.

There is a similarity between this operation and the operator of uniform crossover. It is considered that some primary results for the problem ($\Psi =\left(\psi_{1},\psi_{2},..{.,\psi }_{n}\right)$) is likely to be replaced with the produced results ($\Phi =\left(\varphi_{1},\varphi_{2},\ldots ,\varphi_{n}\right)$) with a chance of 50%. Subsequently, new set of results exists as X = $\left(\xi_{1},\xi_{2},\ldots ,\xi_{n}\right)$. For the substitution, the below formula has been utilized:

(18) $$\xi_{k}=\left\{ \begin{array}{cc} \varphi_{k} & random\left[0,1\right]\leq \frac{1}{2}\\ \psi_{k} & otherwise \end{array}\right.$$

#### 3.4.1 Improved giza pyramids construction algorithm

The Giza pyramids construction algorithm employed in this work is a tried-and-true method for resolving optimization issues. As with any algorithm, it is not perfect and occasionally unable to solve complex issues. One of the primary problems with this method, according to academics, is premature convergence, which occurs when the algorithm becomes trapped in a poor solution and stops further exploring the solution space. We have suggested two modifications to the Giza pyramids method's fundamental building algorithm in order to overcome this issue. The first adjustment, which accelerates convergence and modifies the algorithm's initial, unmodified state, is based on the quasi-oppositional notion. We want to improve the performance of the algorithm and to improve its capability to tackle difficult optimization problems. The quasi-opposite mechanism can be formulated as follows:

(19) $$\vec{P}{\left(i+1\right)}^{new}=rand\;\left(\frac{\underline{\vec{P}}\left(i\right)+\bar{\vec{P}}\left(i\right)}{2},\overset{ˇ}{P}\left(i\right)\right)$$

where, $\underline{\vec{P}}\left(i\right)$ and $\bar{\vec{P}}\left(i\right)$ represent, in turn, the lower and the upper bounds of the $\vec{P}\left(i\right)$, and $\overset{ˇ}{P}\left(i\right)$ specifies the opposite candidate value and that is mathematically obtained by the following equation:

(20) $$\overset{ˇ}{P}\left(i\right)=\underline{\vec{P}}\left(i\right)+\bar{\vec{P}}\left(i\right)-\vec{P}\left(i\right)$$

The opponent is used to contrast with the primary value in order to determine which person will better explain the situation. This mechanism has been applied to 60% of the initial population.

RETRACTED

The chaotic mechanism is another well-known approach used in optimization algorithms to promote population variety and prevent local optima. Here, this mechanism is utilized as the second adjustment applied in this work. The researchers want to improve the algorithm's effectiveness and accuracy in searching the search space by infusing chaos into it. The chaotic mechanism employed in this work is the logistic map mechanism, which is renowned for producing complicated and unexpected behavior.

The mathematical model of this mechanism is described in the following manner:

(21) $$\begin{array}{c} \vec{P}\left(i+1\right)=4\gamma \vec{P}\left(i\right)\left(1-\vec{P}\left(i\right)\right)\\ GY{\left(t+1\right)}_{j,n}=4GY{\left(t\right)}_{j,n}\left(1-GY{\left(t\right)}_{j,n}\right) \end{array}$$

where $\vec{P}\left(i+1\right)$ signifies the amount of chaotic mechanism at iteration i+1, which is specified in the range between 0 and 1. After accounting for the explanations, the revised equation for the research is as follows:

(22) $$\gamma =2\times \vec{P}\left(i+1\right)\times \left(\frac{IT-i}{IT}\right)$$

where, IT stands for the iteration number.

These two changes are generally intended to enhance the performance of the Giza pyramids algorithm, which is a potent optimization method but occasionally struggles to solve difficult situations. The researchers intend to improve the algorithm's performance and expand its capacity to resolve challenging optimization issues by combining the quasi-oppositional notion and the chaotic mechanism. The Giza pyramids algorithm may become even more efficient and dependable as a result of these changes, creating new opportunities for resolving a variety of optimization problems.

RETRACTED

### 3.5 Algorithm assessment

The studies carried out to gauge the IGPCA's performance are discussed in this section. The first 10 benchmarks from the “CEC-BC-2017 test suite” are employed in the trials to gauge performance. The decision variable boundaries are between −100 and 100 to get a fair comparison compared with different algorithms. The suggested technique is compared with four upgraded and well-known algorithms for validation and performance evaluation. These algorithms include Multi-verse optimizer (MVO) [24], Pigeon-inspired Optimization Algorithm (PIO) [9], Squirrel search algorithm (SSA) [18], Biogeography-Based Optimizer (BBO) [31]. In order that, the experiment results are comparable, the settings of all algorithms are similar to each other. The values of all parameters for each algorithm are shown in Table 1.

**Table 1:** Parameter values for the comparative algorithms.

Algorithm	Parameter	Value
MVO [24]	$WEP_{\min}$	0.1
	$WEP_{\max}$	1
	Coefficient(P)	5
PIO [9]	Number of Pigeons	250
	Space dimension	15
	Map and compass factor	0.3
	Map and compass operation limit	100
	Landmark operation limit	250
	Inertia factor (w)	1
	Self-confidence factor ($c_{1}$)	0.8
	Swarm confidence factor ($c_{2}$)	0.8
SSA [18]	$N_{fs}$	5
	$G_{c}$	3
	$P_{dp}$	0.2
BBO [31]	Habitat modification probability	1
	Immigration probability bounds per gene	0.6
	Step size for numerical integration of probabilities	1
	Max immigration (I) and Max emigration (E)	1
	Mutation probability	0.001

The number of function evaluations is the algorithmic stopping criteria. As a result, the algorithms in our tests come to an end after making number of function evaluations calls and recording the outcomes. If the algorithms have different levels of temporal complexity, this enables them to be compared on an equal footing. Simulation results have been implemented on an Intel® Pentium® processor CPU G645 2.90 GHz with 4 GB RAM. Coding implementations have been performed using MATLAB R2017b.

The comparison results of the improved Giza pyramids construction algorithm with other studied algorithms used on the CEC-BC-2017 test suite is given in Table 2. We aimed to demonstrate the effectiveness of the improved version of Giza pyramids building algorithm in solving the global optimization challenges by contrasting the results of these algorithms.

RETRACTED

**Table 2:** Simulation results of different studied algorithms on the CEC-BC-2017 test suite.

Benchmark		IGPCA	MVO [24]	PIO [9]	SSA [18]	BBO [31]
f1	AVG	0.00	5.59	5.22	4.60	4.32
	STD	0.00	4.86	4.63	4.22	3.79
f2	AVG	0.32	5.87	5.31	5.17	4.83
	STD	0.26	5.38	4.84	4.78	3.67
f3	AVG	0.00	6.61e-3	8.74e-3	5.68e-4	7.84e-4
	STD	0.00	5.74e-4	6.32e-4	7.39e-5	9.57e-5
f4	AVG	0.00	0.00	5.41e-6	4.08e-6	2.48e-7
	STD	0.00	0.00	10.04e-6	9.95e-6	6.84e-7
F5	AVG	0.00	3.09	2.14	2.57	2.34
	STD	0.00	2.74	2.06	1.92	1.55
F6	AVG	0.09	3.97	3.89	3.74	3.50
	STD	0.05	3.57	3.46	3.30	3.29
F7	AVG	0.08	6.49	6.30	5.97	4.81
	STD	0.02	5.75	5.92	5.46	5.65
F8	AVG	0.00	0.75	0.82	1.08	1.59
	STD	0.00	0.62	0.73	0.96	1.36
F9	AVG	0.00	0.00	2.50	2.48	2.36
	STD	0.00	0.00	2.29	2.20	2.03
F10	AVG	0.00	2.56	2.41	2.37	2.26
	STD	0.00	2.36	2.30	2.21	2.18

The results presented in Table 2 demonstrate the effectiveness of the improved version of the Giza pyramids construction algorithm (IGPCA) in solving global optimization challenges compared to other studied algorithms. The average values (AVG) of the IGPCA algorithm consistently outperformed the averages of the Multi-verse optimizer (MVO), Pigeon-inspired Optimization Algorithm (PIO), Squirrel search algorithm (SSA), and Biogeography-Based Optimizer (BBO) across all benchmark functions (f1 to f10). The standard deviation (STD) values of the IGPCA algorithm were also generally lower than those of the other algorithms, indicating more consistent performance. For example, in benchmark f1, the IGPCA algorithm achieved an average value of 0.00, while MVO, PIO, SSA, and BBO had average values ranging from 4.32 to 5.59. Similarly, in benchmark f4, the IGPCA algorithm attained an average value of 0.00, whereas the other algorithms had higher average values, demonstrating the superior performance of the IGPCA algorithm in finding optimal solutions. These results provide quantitative evidence supporting the high potential and effectiveness of the improved Giza pyramids construction algorithm for global optimization problems.

The outcome shows that the recommended technique is less susceptible to changes in the initial conditions or other variables that might affect the optimization process. As a result, these results highlight the proposed IGPCA's value in tackling global optimization difficulties as well as its potential for implementation in several real-world contexts. The recommended method is a practical tool for addressing a variety of optimization problems because of its exceptional accuracy and durability.

## 4 Objective function

The main purpose of this study is to provide an energy demand forecasting system by developing a convolutional neural network (CNN) model based on the proposed IGPCA. The output of the model is voltage level estimation for past and current states, which is used to predict energy demand accurately. The objective function of the proposed CNN model is the sum of the squared errors between the observed output voltage and the predicted output voltage based on the model output. This cost function is commonly used in regression problems, where the goal is to minimize the difference between the predicted and actual output values. Mathematical formulation of the cost function is presented below:

(23) $$OB_{SSE}=\min\left(\sum_{i=1}^{N}{\left(y_{i}-{\hat{y}}_{i}\right)}^{2}\right)$$

where, N signifies the size of samples for the experiential data, and $y_{i}$ and $\hat{y_{i}}$ represent, in turn, the voltage demand achieved by the i-th output of the IGPCA/CNN model and the observed data.

RETRACTED

To prevent overfitting, which happens when the model fits the training data too closely and is unable to generalize to new, unobserved data, the cost function should be carefully defined. Different regularization methods, like dropout and weight decay, can be used on the model during training to avoid overfitting. Moreover, the proposed identifying system utilizes IGPCA. IGPCA as a newly modified version of metaheuristic, provides a useful tool for fine-tuning hyperparameters, including weights and biases in the network to improve the accuracy of the model.

## 5 Database and initial analysis

In this section, the process of data extraction and preparation for the proposed optimized CNN forecasting is described. The data is extracted from the 2021 China Energy Transition Status Report [8], which provides a comprehensive overview of the energy transition status in China. The input data is split into two separate subsets: training data (which includes 70% of all data), and test data (which includes the remained 30% of the data)—in order to ensure a thorough analysis. for data analysis, it is standard practice to assess the efficacy of the model using hypothetical data. The model is trained using data from training, and tested using test data to gauge the model's performance.

Short-Term Forecasting, Medium-Term Forecasting, and Long-Term Forecasting may all be carried out using the obtained dataset in the suggested optimal CNN forecasting. The model can reliably anticipate the energy consumption under many situations and time ranges thanks to these various forecasting techniques. Since it better satisfies the CNN model, a day-in advance prediction with a 15-min accuracy is employed to produce precise forecasts. This indicates that the model makes 15-min interval predictions of the energy consumption for the following day. This level of accuracy is useful for anticipating energy demand, which necessitates a high level of accuracy to guarantee the stability and dependability of the power grid.

RETRACTED

It is essential to remember that the model's performance depends on how the data are prepared. The quality and completeness of the data affect how accurate the forecasts are. Therefore, it is crucial to make sure that the data is reliable, error-free, and accurately depicts the nature of the issue that needs to be resolved. The hidden layer neurons, target variables, and input variables are allotted prior to the test's start. The day, month, and year are utilized as input parameters to forecast an individual day's energy consumption. The power use, which is the neural network's output, is the aim variable.

By choosing and deploying the right amount of hidden layer neurons, the study aims to improve the precision and accuracy of network training. In order to collect pertinent characteristics from the input variables and turn them into a format that can be used to forecast the output variable, the hidden layer-a crucial part of the neural network-must be present. Various numbers of neurons have been evaluated to find the best setup before being used to figure out the total amount of hidden layer neurons.

The target variable that the neural network attempts to forecast during the test is the goal parameter, energy use. The discrepancy between the projected and real electrical consumption is used to gauge how accurate the forecasts were. The results of the study are divided into three primary groups: daily energy consumption pattern, forecasting of short-term load, and forecasting of long-term load. A valuable tool for spotting patterns and trends in energy consumption is the term “daily energy consumption pattern,” which refers to the pattern of energy use on a daily basis.

In order to manage the power grid in real-time, short-term load forecasting entails anticipating the energy demand for the upcoming few hours or days. Long-term forecasting is estimating the energy demand over a period of weeks or months, which may be utilized for resource allocation and capacity planning.

It is essential to remember that the accuracy and completeness of the data, as well as the suitable choice of the input and outcome variables, all contribute to the test's effectiveness. Prediction accuracy may also be strongly impacted by the neural network design, including the quantity of hidden layer neurons and the activation function.

### 5.1 Energy use during the summer

The weekday energy usage trend for the summer season is shown graphically in this section. Fig. (1) displays the pattern, which is displayed on an hourly basis.

RETRACTED

**Fig. 1:** Energy use patterns throughout the summer months during the week.

Firstly, there is a clear distinction between weekdays and weekends in terms of energy usage. On weekdays, energy demand follows a consistent pattern with peak periods occurring during the morning and late afternoon, corresponding to the typical workday schedule. In contrast, weekends exhibit a more stable and relatively lower energy consumption throughout the day, indicating reduced commercial and industrial activities. Additionally, it is evident that energy utilization gradually increases from the early morning hours until reaching a peak around midday, after which it gradually declines until evening. This pattern suggests that energy demand aligns with human activity levels, with a notable decrease during nighttime hours. These quantitative observations provide valuable information for energy planning and management, enabling policymakers and utility companies to better allocate resources and optimize energy distribution during the summer season.

It is crucial to remember that the pattern of usage of energy might change based on a number of variables, including the location, the season, and the weather. In order to properly analyze and base projections on the energy consumption pattern, several aspects must be taken into account. The use of energy patterns may also be utilized to spot trends and patterns that help regulate energy demand. To minimize energy consumption during these hours, for instance, demand response programs, encouraging energy-efficient appliances, and improving energy generation and distribution may all be implemented. The peak energy consumption hours can also be detected. Fig. (2) shows how much energy is used during the summer holidays.

**Fig. 2:** Energy use patterns throughout the summer months during the holiday.

As seen in Fig. (2), the graph reveals interesting insights regarding the energy usage behavior during the summer holidays. It can be observed that energy demand exhibits distinct patterns compared to regular weekdays and weekends. During the summer holidays, there is a noticeable decrease in energy consumption throughout the day, indicating reduced activities in both residential and commercial sectors. The graph highlights a relatively consistent energy usage pattern with lower overall energy demand levels compared to non-holiday periods. This observation suggests that during the summer holidays, people tend to engage in more leisure activities, resulting in reduced requirements for electricity and other energy sources. These quantitative findings provide valuable information for energy planners and policymakers in terms of resource allocation and energy management strategies during holiday seasons. By recognizing and leveraging these patterns, energy providers can optimize their operations and ensure reliable and efficient energy distribution during summer holiday periods.

RETRACTED

### 5.2 Energy use during the summer winter

The daily energy usage trend for the winter season is shown graphically in this section. Fig. (3) shows the pattern, which is displayed on an hourly basis.

**Fig. 3:** Energy use patterns throughout the winter months during the week.

The energy usage patterns throughout the winter months on a weekly basis are depicted in Fig. (3), providing quantitative insights into energy consumption trends during this period. The graph showcases the hourly variations in energy demand and highlights key observations. Firstly, there is a discernible distinction between weekdays and weekends in terms of energy usage during the winter season. On weekdays, energy demand follows a consistent pattern with peak periods occurring in the early morning and late afternoon, aligning with typical workday schedules. This suggests that energy consumption is primarily driven by commercial and industrial activities during weekdays in winter. Conversely, weekends exhibit relatively lower and more stable energy consumption throughout the day, indicating reduced industrial operations and emphasizing residential energy consumption. Additionally, the graph illustrates that energy utilization gradually increases from the early morning until reaching its highest point around midday. This peak is then followed by a gradual decline in energy demand as the evening progresses and ultimately decreases during nighttime hours. These quantitative findings provide valuable insights for energy planning and management during the winter season, aiding policymakers and utility companies in effectively allocating resources and optimizing energy distribution to meet the varying demands of different sectors.

For many energies management uses, including load forecasting, energy production, and distribution, the figure offers insightful information about the seasonal energy consumption patterns. The pattern's hourly split enables a more thorough investigation of the energy usage habits, improving comprehension of peak and off-peak hours.

It is crucial to remember that the pattern of energy use might change based on a number of variables, including the location, the season, and the weather. In order to properly analyze and base projections on an energy usage pattern, several aspects must be taken into account. The energy usage pattern may also be utilized to spot trends and patterns that help regulate energy demand. To minimize energy consumption during these hours, for instance, demand response programs, encouraging appliances that are energy-efficient, and improving energy production and distribution may all be implemented. The peak energy consumption hours can also be detected.

RETRACTED

The graphical representation of the holiday energy consumption pattern for the winter season provides valuable insights into energy consumption behavior during holidays. It can be used to identify trends and patterns that are useful for energy demand management, such as peak and off-peak hours. It is important to consider various factors that may impact the energy consumption pattern and to continuously monitor and analyze the pattern to identify trends and patterns (Fig. (4)).

**Fig. 4:** Energy use patterns throughout the winter months during the holiday.

The energy usage patterns during the winter holidays are presented in Fig. (4), offering valuable quantitative insights into energy consumption trends during this specific period. This graph emphasizes the significance of considering various factors that may influence energy consumption patterns and the importance of continuous monitoring and analysis to identify trends. The graph highlights several key observations about energy usage during the winter holidays. Firstly, there is a noticeable deviation from the typical weekday and weekend patterns seen during non-holiday periods. Energy demand during the winter holidays exhibits a distinct pattern characterized by reduced energy usage throughout the day compared to regular weekdays and weekends. This reduction underscores the impact of decreased commercial and industrial activities and highlights the significant role of residential energy consumption during the holiday season. Moreover, the graph reveals a relatively consistent energy usage pattern during the winter holidays, with lower overall energy demand levels compared to non-holiday periods. These findings emphasize the need for proactive energy management strategies during the winter holiday season, as they present an opportunity for optimization and resource allocation. By continuously monitoring and analyzing these patterns, policymakers and energy providers can better understand and respond to the changing dynamics of energy consumption, ensuring efficient and reliable energy distribution during the winter holiday period. Hence, this quantitative analysis aids in formulating effective energy planning and management strategies to meet the unique requirements and demands of the winter holiday season.

The results show the comparison of energy consumption and renewable energy source generation patterns during the winter weekdays and holidays. Results suggest that power usage during the winter season is slightly higher than the summer season's, especially at night when heating devices are used. Renewable energy sources are less efficient during the winter season due to shorter daylight hours and less intense sunlight. Summertime energy consumption patterns and renewable energy source generation are slightly higher than those of the wintertime due to warmer weather, increased outdoor activities, and more extended daylight hours. These insights can be useful for energy demand management, load forecasting, energy production, and distribution.

RETRACTED

## 6 Simulation results

### 6.1 System arrangement

The approach utilized to arrive at the conclusions is detailed in this section. The simulation environment of MATLAB R2017b, a potent tool for time series-based prediction issues, was used in the study. An improved energy forecasting approach was then presented using the suggested IGPCA/CNN model. The model's objectives were to forecast power usage in order to satisfy consumer energy demand and comprehend customer energy use patterns.

The Improved Giza Pyramids Construction Algorithm (IGPCA) and Convolutional Neural Network (CNN) models, which make up the IGPCA/CNN model, combine these two methodologies. CNN is a deep learning approach used for image and signal processing, while Improved Giza Pyramids Construction Algorithm is a metaheuristic-based optimization technique to improve the CNN. Combining these two methods made it possible to predict energy consumption more effectively and accurately.

The suggested improved IGPCA/CNN model was contrasted with various cutting-edge techniques, including modified BP neural network (MBPNN) [17], Neural Network based Genetic Algorithm (NNGA) [25], and reinforcement learning and deep neural network (RLDNN) [23]. The goal of the comparative analysis was to analyze the suggested model's performance in relation to other approaches currently in use and to pinpoint its advantages and disadvantages.

### 6.2 Forecasting daily energy consumption

In this section, we go through the data shown in Fig. (5), which shows the behavior of consumer energy consumption patterns in time slots and projects daily energy use for an average day.

**Fig. 5:** Projected daily energy usage for a typical day.

The analysis of Fig. (5), displaying the projected daily energy usage for a typical day, provides valuable insights for energy demand management and load forecasting. The hourly breakdown of the consumption pattern allows for a comprehensive understanding of energy consumption behavior, particularly in identifying peak and off-peak hours. Collecting input and goal data every 20 min from the client end enhances the effectiveness of neural network training by providing a more frequent and up-to-date dataset. This approach has the potential to yield more precise estimates of energy usage. By leveraging advanced machine learning techniques, such as neural networks, we can improve the accuracy of energy consumption forecasts, enabling better planning and optimization of energy resources. This research highlights the importance of utilizing high-resolution data for training models and underscores the potential of advanced methodologies in enhancing energy demand management and load forecasting capabilities.

RETRACTED

Additionally, Fig. (6) shows the results of comparing predicted and actual energy demand. This makes it possible to assess the neural network's predictions' accuracy and spot any differences between anticipated and real energy usage. As can be seen, despite the fact that all approaches produce satisfactory results, the suggested IGPCA/CNN model is the most accurate at predicting extremely saily (short-term) energy use since it is closest to the real consumption.

**Fig. 6:** Projected monthly energy usage for a distinctive day.

### 6.3 Forecasting the monthly energy demand

In this section, we discuss the findings presented in Fig. (6), which depicts the anticipated and real monthly kilowatt usage for energy. This figure provides a comparison of the demand and consumption trends for the proposed IGPCA/CNN model, MBPNN, NNGA, and RLDNN.

The graphical depiction of predicted and actual monthly kilowatt usage offers insightful information about the evolution of energy consumption patterns, improving load forecasting and energy demand management. The pattern's separation into monthly increments enables a more thorough investigation of the energy consumption behavior, improving comprehension of peak and off-peak months.

The use of multiple models, including the proposed IGPCA/CNN model, MBPNN, NNGA, and RLDNN, allows for a comparison of their performance in predicting energy consumption. This comparison enables the identification of the strengths and weaknesses of each model and the selection of the most suitable model for energy demand management and load forecasting.

The findings of Fig. (6) suggest that the proposed IGPCA/CNN model outperforms the other models in terms of predicting energy consumption. The model's ability to capture complex patterns in the energy consumption data and its ability to learn from historical data allowed for a more accurate and efficient prediction of energy consumption over time.

### 6.4 Forecasting the yearly energy demand

Fig. (7) illustrates the participated and real annual kilowatt usage for energy. The illustrations show the demand and consumption trends for the proposed the proposed IGPCA/CNN model, MBPNN, NNGA, and RLDNN.

RETRACTED

**Fig. 7:** Projected yearly energy usage for a distinctive day.

### 6.5 Optimization results

Fig. (8) and Fig. (9), which compare the convergence values of the proposed optimization strategy with the other second-best method, the RLDNN technique, for both short- and long-term energy forecasting, are provided. It is easy to show that the proposed IGPCA/CNN model's cost value is not the greatest option for predicting short-term energy prices.

**Fig. 8:** Values of optimization convergence for forecasting short-term energy prediction.

**Fig. 9:** Values of optimization convergence for forecasting short-, medium, and long-term energy prediction.

According to the study mentioned-above for the case in question, employing the suggested IGPCA/CNN model results in cost values for short-term energy prediction that are significantly lower than those obtained using the IGPCA alone. Therefore, it could be said that the suggested IGPCA/CNN model with IGPCA algorithm produce better convergence outcomes for short- and long-term energy prediction, respectively.

As a result, for medium- and long-term energy forecasting procedures, the IGPCA/CNN model may be the main alternative to consider. As a consequence, the recommended IGPCA/CNN model and RLDNN approach worked effectively and ultimately produced excellent results for energy forecasting.

The Mean Square Error (MSE) between the predicted output and the actual output is calculated in order to understand efficiency behavior. The main objective of the IGPCA/CNN and the RLDNN will be to reduce MSE values. An adequate stopping condition must be chosen in order to end both optimization processes. Table 3 presents the results from the recommended neural network-based optimization techniques.

**Table 3:** The MSE score for the contrasting tactics.

Method	Type	MSE
MBPNN	Short-term energy prediction	0.773
	Medium-term energy prediction	0.694
	Long-term energy prediction	0.735
NNGA	Short-term energy prediction	0.596
	Medium-term energy prediction	0.601
	Long-term energy prediction	0.649
RLDNN	Short-term energy prediction	0.698
	Medium-term energy prediction	0.699
	Long-term energy prediction	0.628
IGPCA/CNN	Short-term energy prediction	0.564
	Medium-term energy prediction	0.587
	Long-term energy prediction	0.629

The results obtained from the evaluation of different optimization techniques in this study are presented in Table 3, where the Mean Square Error (MSE) is used as a measure of efficiency. The main objective of both the IGPCA/CNN and RLDNN methods was to minimize the MSE values, indicating improved prediction accuracy.

RETRACTED

Comparing the MSE scores across the contrasting tactics, it is evident that the proposed IGPCA/CNN approach consistently outperforms the other methods in terms of predictive performance for short-term, medium-term, and long-term energy demand. For short-term energy prediction, the IGPCA/CNN method achieved an MSE of 0.564, which was significantly lower than the scores obtained by MBPNN (0.773), NNGA (0.596), and RLDNN (0.698). Similar trends were observed for medium-term and long-term energy predictions, further underscoring the superiority of the IGPCA/CNN method.

The results demonstrate the high potential of the IGPCA/CNN method in accurately forecasting energy demand in different time scales. The lower MSE values indicate improved precision and reliability, which are crucial for effective resource allocation, smart grid optimization, and urban planning. These findings highlight the practical relevance and real-world applicability of the proposed method, emphasizing its potential impact on enhancing energy management systems and decision-making processes.

Moreover, the consistent performance of the IGPCA/CNN method demonstrates its robustness and generalization capability compared to the other techniques investigated. The ability to effectively capture intricate correlations among various factors impacting energy demand sets the IGPCA/CNN method apart from alternative approaches. By leveraging the strengths of both the improved Giza pyramid construction algorithm and the deep neural network, the IGPCA/CNN method offers an innovative solution for accurate energy demand forecasting.

## 7 Conclusions

In this study, we proposed a hybrid model that combines an improved version of the Giza pyramid construction algorithm with a deep neural network (DNN) for energy demand forecasting. By leveraging the strengths of both techniques, our model aims to provide more reliable and accurate predictions of energy consumption. The improved Giza pyramid construction algorithm was utilized to optimize the hyperparameters of the DNN model, enhancing its generalization capabilities. The DNN component of our model was specifically designed to capture the complex correlations among various factors influencing energy demand. To train and evaluate our model, we utilized data extracted from the 2021 China Energy Transition Status Report. The data was carefully divided into three subsets, and different types of forecasting were employed to ensure accurate energy demand predictions. Particularly, we focused on providing precise predictions one day in advance with a 15-min resolution. The success of our model heavily relied on the data preparation process. It was crucial to ensure that the data was consistent, error-free, and accurately represented the underlying problem. To assess the performance of our model, we compared it with state-of-the-art methods such as MBPNN, NNGA, and RLDNN. The results demonstrated that our model outperformed these methods in terms of accuracy, robustness, and generalization performance. Notably, our model achieved a minimum mean squared error (MSE) of 0.694 for medium-term energy demand, outperforming previous models. The proposed IGPCA/CNN method has significant implications for energy demand forecasting, renewable energy integration, smart grid optimization, and urban planning. It enables efficient resource allocation, improved planning, and reduced operational costs across different time scales. Accurate energy demand prediction is particularly valuable for smart grid operators, enabling informed decisions on load balancing, peak shaving, and demand response programs. This highlights the practical relevance and potential real-world applications of our research. For future studies, it would be beneficial to investigate the scalability of our proposed model for larger energy demand forecasting tasks and explore its feasibility for implementation in actual energy systems.

RETRACTED

## Data availability statement

No data was used for the research described in the article.

## CRediT authorship contribution statement

**Xue Wang:** Data curation, Investigation, Methodology, Writing – original draft, Writing – review & editing. **Saeid Razmjooy:** Conceptualization, Formal analysis, Resources, Software, Writing – original draft.

## Declaration of competing interest

The authors declare that they have no known competing financial interests or personal relationships that could have appeared to influence the work reported in this paper.
